# A Comparative Study of ARHI Imprinted Gene Detection and Fine-Needle Aspiration Cytology in the Differential Diagnosis of Benign and Malignant Thyroid Nodules

This article has been retracted.

**DOI:** 10.1089/gtmb.2019.0028

**Published:** 2019-09-12

**Authors:** Dazhong Zou, Chengwei Wu, Jixuan Miao, Qing Shao, Wenlong Huang, Jianda Huang, Guihua Wu, Qing Zhang

**Affiliations:** ^1^ Department of Ultrasonography, The Jiangyin Clinical College of Xuzhou Medical University, Jiangyin, China.; ^2^ Department of Ultrasonography, Suzhou Wuzhong People's Hospital, Suzhou, China.

**Keywords:** ARHI, imprinted gene, thyroid nodule, fine-needle aspiration cytology

## Abstract

***Aims:*** To compare fine-needle aspiration cytology (FNAC) with imprinted gene detection in the differential diagnosis of benign and malignant thyroid nodules.

***Methods:*** A total of 34 patients (35 cases of thyroid nodules) were examined using fine-needle puncture biopsy under ultrasound guidance, and the biopsy tissues were examined by cytologic examination and imprinted gene detection. Combined with postoperative pathology and follow-up results, the diagnostic value and consistency of the two methods were analyzed and compared.

***Results:*** The detection of benign and malignant thyroid nodules by ARHI imprinted gene had a high consistency with FNAC, and ARHI imprinted gene detection had a higher detection rate, sensitivity, and accuracy.

***Conclusions:*** Imprinted gene detection has high accuracy and sensitivity in the differential diagnosis of benign and malignant thyroid nodules. It provides a scientific reference for clinical treatment and should be incorporated into diagnostic protocols for thyroid tumor.

## Introduction

Thyroid nodule is a common endocrine disease, which is often without obvious clinical symptoms; the detection rate of its ultrasound screening is as high as 20–76% (Wong *et al.*, 2018). The judgment of benign and malignant of thyroid nodule is the core to determine the subsequent treatment plan. Ultrasound-guided fine-needle aspiration cytology (FNAC) is an important diagnostic method for preoperative assessment of thyroid nodules, which was first developed in developed countries in the 1980s and has been widely used since then; however, the results of FNAC with no diagnostic value or unclear significance still cause distress to the clinical management of such patients (Collins *et al.*, 2015; Park *et al.*, 2018).

In recent years, with the rapid development of tumor molecular pathologic diagnosis, the role of imprinted genes in human genetic diseases, especially in tumorigenesis, has been given increasing attention (Lee *et al.*, 2017; Menoni *et al.*, 2017). From the perspective of tumorigenesis, the imprinted gene is equivalent to a functional haploid, which requires only one mutation to inactivate or activate the gene, thereby increasing the susceptibility of tumors (Muthu *et al.*, 2015). Unlike other proto-oncogenes of the Kirsten rat sarcoma viral oncogene homolog (KRAS) family, ARHI at 1p31 was the first maternal-imprinted tumor suppressor gene to be discovered. Studies have reported that ARHI can lose imprinting or methylation in most ovarian carcinoma, breast cancer, pancreatic cancer, thyroid cancer, and brain tumor (Li *et al.*, 2014; Lu *et al.*, 2014; Washington *et al.*, 2015; Damaschke *et al.*, 2017).

*In situ* detection of imprinted gene is an advanced detection technology based on epigenetics theory and *in situ* hybridization technology, which the expression, deletion, and copy number variation (CNV) of ARHI imprinted genes in the samples of cancer patients can be visually and accurately observed and detected (Lee *et al.*, 2017). At present, this technique is still in the exploratory stage of clinical application, and the comparative study between the detection results and the pathological results (considered as the “gold standard”) has been rarely reported. Therefore, the present study was designed to compare the value of FNAC cytology results with that of imprinted gene detection in the differential diagnosis of benign and malignant thyroid nodules.

## Materials and Methods

### Patients

A total of 34 patients with thyroid nodules (35 cases of thyroid nodules) admitted to the department of breast and thyroid surgery of Jiangyin People's Hospital from January to December 2017 consecutively and examined by ultrasound-guided FNAC were selected in this research.

Inclusion criteria are as follows: patients with thyroid nodules had the following two or more suspicious malignant ultrasound image characteristics (Wong *et al.*, 2018): (1) presence of sand-like calcification; (2) thyroid nodules in low echo level; (3) abundant blood flow in nodules; (4) unclear nodule boundaries and infiltration to the surrounding area; (5) irregular nodule morphology; (6) the anteroposterior diameters of transverse section were larger than the left and right diameter; and (7) enlargement of peripheral lymph nodes.

Exclusion criteria are as follows: (1) patients with history of bleeding for unknown causes; (2) patients with bleeding tendency (activation time of partial thrombin was 10 s longer than the upper limit of normal range, prothrombin time was 3–5 s longer than the upper limit of normal range, fibrinogen level was less than 1 g/L, platelet count was less than 50,000/mm,^3^ and the aggregation function was poor); (3) patients with severe hypertension (systolic blood pressure more than 180 mmHg); and (4) patients who were unwilling to cooperate.

Ultrasound-guided FNAC and imprinted gene detection were performed in all selected patients. Before examination, the method, purpose, precautions, and possible complications of puncture were explained to the patients in detail. All patients signed the informed consent. This study was approved by the Ethics Committee of Jiangyin People's Hospital.

### Methods

Apparatuses and reagents were as follows: MyLab TWICE Color Ultrasonic Diagnostic Apparatus (Esaote Company, Italy) with the probe frequency at 5–12 MHz; the apparatus used for needle aspiration was the disposable sterile injection needle PCT-B18*200 (BD Company) and 10 mL disposable syringe; 10 mL cell lysate (Lisen Imprinted Diagnostic Technology Wuxi Co., Ltd.).

(1) Routine electrocardiogram, blood routine, all items of coagulation, liver function, kidney function, five items of hepatitis B, syphilis, AIDS, hepatitis c, and thyroid function (FT3, FT4, and TSH) were examined before puncture biopsy. The room was disinfected, medicines such as lidocaine, hemostatic agent, and dexamethasone were prepared for use, and routine ultrasound examination was conducted before puncture. The size and blood flow of the nodules were evaluated by color Doppler, and the optimal puncture path was determined according to the evaluation.

(2) The puncture process was performed by two doctors of the department of ultrasound and intervention. Patient was in a supine position with the shoulder raised and the neck completely exposed, then the patient was sterilized, without anesthesia. Ultrasound was used to observe the needle insertion point in real time, and the angle was adjusted as the needle was inserted until the tip reached the substantial part of the nodule. Two to three needles were punctured for each nodule, and each needle was punctured for three to five times in multiple directions within the nodule, and negative pressure suction was performed. The sample obtained by puncture was quickly smeared after the needle was removed. All smear specimens were diagnosed by the same pathologist. After puncture, the patient was instructed to gently press the puncture site for 15 min to stop bleeding, and could leave after 30 min if there was no discomfort.

The cytopathological diagnosis of FNAC followed the guideline ATA 2015: (1) specimens those were undiagnosed or unsatisfactory, (2) benign lesions, (3) inconclusive atypical cell lesions or follicular lesions, (4) follicular or suspicious follicular tumors, (5) suspicious tumors, and (6) malignant tumors (Haugen *et al.*, 2016). Benign lesions were regarded as negative, and suspicious malignant and malignant were regarded as positive (Table 1).

**Table 1.** Criteria for Fine-Needle Aspiration Cytology Cytopathological Diagnosis Results

*Cytopathological diagnosis results*	*Criteria*
Undiagnosed	The specimens were poorly sampled, and there were not enough cellular components in the smear to make cytological diagnosis
Benign lesions	Diagnosis of nonneoplastic disease
Suspicious malignant	Follicular tumors and eosinophilic tumors, as well as some cytological features suggestive of malignant, but could not be diagnosed as malignant lesions
Malignant	Malignant diagnosis that could be confirmed, including papillary adenocarcinoma, medullary carcinoma, undifferentiated carcinoma, lymphoma, and metastatic carcinoma

The other sample was rinsed in an EP tube containing 10 mL of cell lysate. After the cap was tightened, the sample was mailed to Lisen Imprinted Gene Company of Wuxi. Quantitative analysis was performed according to the total expression amount of ARHI imprinted gene, loss of imprinting (LOI), and the nucleus proportion with CNV in the thyroid tissue or puncture cell samples, and the benign and malignant tumors were evaluated and divided into four categories: (1) undiagnosed, (2) benign, (3) malignant potential (category V), and (4) malignant (category VI). The benign was regarded as negative, and the malignant and malignant potential were regarded as positive.

(3) Surgical treatment was performed and pathological types were recorded for patients with positive FNAC, ARHI imprinted gene detection showed positive, presence of compression symptoms or nodule enlargement and ultrasonic characteristics change during short-term follow-up. Otherwise, long-term follow-up was conducted for 6 months. During the long-term follow-up, tissues whose reexamination results of FNAC were still negative and no enlargement or change in nature of nodules found by ultrasound examination were considered as benign.

### Statistical analysis

SPSS 23.0 software was used for data analysis. The continuous variables were presented as ${\overline x}$ ± SD, and *t*-test was used for comparison between groups. The categorical variables were expressed by percentage (%), and *χ*^2^ test was used for comparison between groups. The consistency test of Kappa analysis and diagnosis was performed by using FNAC and ARHI imprinted gene detection. There is a significant difference at *p* < 0.05. The detection rate, sensitivity, specificity, positive predictive value, negative predictive value, and accuracy of the two methods were calculated by referring to the surgical pathology and follow-up results. Receiver operating characteristic (ROC) curve was constructed to analyze the differences in area under curve (AUC), and the diagnostic value of the two methods was evaluated.

## Results

### Clinical characteristics

A total of 34 patients were enrolled in the study, including 6 males and 28 females (44.3 ± 26.1 years). All patients underwent ultrasound, cytological classification, and imprinted gene detection. Finally, 29 patients (30 cases of thyroid nodules) received surgery, and another 5 patients were diagnosed as benign after follow-up. Twenty-two of the 30 cases of nodular surgery were malignant, and the remaining 8 were benign. The age of malignant patients was younger than that of benign patients, and the nodule size of malignant patients was smaller than that of benign patients (*p* < 0.05; Table 2).

**Table 2.** Clinical Characteristics of the Subjects and Nodules

*Group*	*Number (male/female)*	*Age (year)*	*Diameter of nodules (cm)*
Benign	13 (2/11)	46.7 ± 8.9	1.43 ± 0.41
Malignant	22 (4/18)	36.4 ± 9.4	1.10 ± 0. 32
*χ*^2^	0.045	3.164	2.848
*p*	0.832	0.003	0.008

### Classification results and consistency of the two methods

Among the 35 cases of thyroid nodules in 34 patients, there were 15 cases of malignant, 5 cases of suspicious malignant (Fig. 1), 10 cases of benign lesions, and 5 cases of undiagnosed diagnosed by FNAC; meanwhile, there were 18 cases of malignant (Fig. 2), 7 cases of malignant potential, 7 cases of benign, and 3 cases of undiagnosed detected by ARHI imprinted gene (Tables 3–5). Statistical analysis of the consistency test of the two methods indicated that the imprinted gene detection was alignment with FNAC in the diagnosis of benign and malignant thyroid (Kappa = 0.707, *p* = 0.000).

**FIG. 1.** Thyroid FNA smear cytology examination. A small number of proliferating follicular epithelial cells were seen in the sample, which were arranged in a follicular pattern with enlarged nucleus and deepened staining. The examination result was inconclusive follicular lesions. FNA, fine needle aspiration.

**FIG. 2.** Thyroid ARHI imprinted gene detection. Two or more staining markers appeared in multiple nucleus in the sample, indicating that LOI and CNV, and the genetic detection result was malignant. LOI, loss of imprinting; CNV, copy number variation.

**Table 3.** Comparison of Fine-Needle Aspiration Cytology and ARHI Imprinted Gene Detection Results (n)

*ARHI imprinted gene detection FNAC*	*Undiagnosed*	*Benign lesions*	*Malignant potential*	*Malignant*	*Total*
Undiagnosed	3	0	2	0	5
Benign	0	7	2	1	10
Malignant potential	0	0	3	2	5
Malignant	0	0	0	15	15
Total	3	7	7	18	35

FNAC, fine-needle aspiration cytology.

**Table 4.** Fine-Needle Aspiration Cytology and Clinical Diagnosis Results (n)

*Detection method*	*Clinical diagnosis of malignant*			*Clinical diagnosis of benign*		
	*Positive*	*Negative*	*Undiagnosed*	*Positive*	*Negative*	*Undiagnosed*
FNAC	18	2	2	2	8	3

**Table 5.** Comparison of ARHI Imprinted Gene Detection and Clinical Diagnosis Results (n)

*Detection method*	*Clinical diagnosis of malignant*			*Clinical diagnosis of benign*		
	*Positive*	*Negative*	*Undiagnosed*	*Positive*	*Negative*	*Undiagnosed*
ARHI imprinted gene detection	22	0	0	3	7	3

### Postoperative histopathological classification results

Of the 22 cases of malignant diagnosed by postoperative pathology, there were 21 cases of papillary thyroid carcinoma (PTC), 1 case of follicular thyroid carcinoma (FTC), while the remaining 8 benign nodules included 5 cases of multinodular goiter (MNG), 2 cases of Hashimoto's thyroiditis, and 1 case of subacute thyroiditis (Fig. 3).

**FIG. 3.** Postoperative histopathological classification results. PTC, papillary thyroid carcinoma; FTC, follicular thyroid carcinoma; MNG, multinodular goiter; HT, Hashimoto's thyroiditis; SAT, subacute thyroiditis.

ARHI imprinted gene malignancy was detected in 18 cases of nodules, and confirmed by postoperative pathology, 16 cases were PTC, 1 case was FTC, and 1 case was MNG. Of the seven cases of nodules with potential malignant of imprinted ARHI gene, with postoperative pathology, five cases were diagnosed as PTC, one case was diagnosed as MNG, and one case with repeated FNAC and ultrasonic follow-up was diagnosed as benign.

### Comparison of the values of ARHI imprinted gene detection and cytological pathology diagnosis of category III and IV thyroid nodules

Category III is likely to be benign disease; category IV is regarded as abnormal, and the possibility of malignant lesions cannot be ruled out, so further biopsy is needed to make it clear. Apart from the undiagnosed cases, benign lesions in FNAC and ARHI imprinted gene detection results were considered negative, while suspicious malignant (malignant potential) and malignant were considered as positive. The detection rate, sensitivity, specificity, positive predictive value, negative predictive value, and accuracy of FNAC calculated by referring to surgical pathology and follow-up results were 85.7%, 90.0%, 80.0%, 90.0%, 80.0%, and 86.7%, respectively. The detection rate, sensitivity, specificity, positive predictive value, negative predictive value, and accuracy of ARHI imprinted gene detection were 91.4%, 100.0%, 70.0%, 88.0%, 100.0%, and 90.6%, respectively. The detection rate, sensitivity, negative predictive value, and accuracy of imprinted gene detection were higher than those by FNAC (Table 6 and Fig. 4). The AUC values of the ROC curve in both methods were 0.850.

**FIG. 4.** ROC curves of FNAC and ARHI imprinted gene detection. ROC, receiver operating characteristic; FNAC, fine-needle aspiration cytology.

**Table 6.** Comparison of Diagnosis Values of the Two Methods (%)

*Methods*	*Detection rate*	*Sensitivity*	*Specificity*	*Positive predictive value*	*Negative predictive value*	*Accuracy*
FNAC	85.7	90.0	80.0	90.0	80.0	86.7
ARHI imprinted gene detection	91.4	100.0	70.0	88.0	100.0	90.6

## Discussion

Ultrasound examination is noninvasive and nonradiative and is an important method to differentiate the benign and malignant thyroid nodules. The morphology, boundary, capsule, echodensity, microcalcification, and blood supply of thyroid nodules are important factors to judge the benign and malignant of thyroid nodules. However, this method can be influenced by the clinical experience of the ultrasound physician.

Thyroid FNAC is the most widely used preoperative evaluation test at present, with high sensitivity and specificity (Ucler *et al.*, 2015). In this study, the sensitivity and specificity of FNAC results were 90% and 80%, respectively, which were consistent with the sensitivity of 65–98% (median 83%) and specificity of 72–100% reported in previous literature (Lee *et al.*, 2017; Ha *et al.*, 2018). However, the proportion of specimens without diagnostic value reached 14.3%, exceeding the recommended upper limit (7%). The reasons for this result included (1) the technical level of thyroid puncture and the quality of cytopathology slides were not good; (2) the professional skill varied among pathologists; and (3) the nature of thyroid lesions was different, such as when the lesion was cystic, the cystic fluid component that was often seen by puncture cell components were too few (Rong *et al.*, 2016).

Imprinted gene is a ubiquitous epigenetic phenomenon, an important regulatory mechanism of gene expression, and a biomarker at the molecular level. ARHI at 1p31 is the first maternal-imprinted tumor suppressor gene to be discovered; it has 50–60% amino acid homology with KRAS, but performs the opposite function, inhibiting cell growth, movement, and invasion (Li *et al.*, 2014). The changes of imprinted genes occurs in the early stage of tumor development, and the imprinted genes changed before the changes of cell morphology. Therefore, the greatest highlight of imprinted diagnosis is its sensitivity to early tumors. The results of this study showed that the sensitivity of ARHI imprinted gene was 100%, which was consistent with the theory. However, the specificity of imprinted gene detection was only 70%, and for the results of ARHI imprinted gene detection of thyroid nodules in three cases clinically diagnosed as benign (two cases were confirmed by surgery), two cases were potential malignant and 1 case was malignant. The reasons might be as follows: (1) as changes in molecular level, changes in the status of ARHI imprinted gene were not always the result of the development of histopathological cancer and (2) the change of ARHI imprinted gene status was an early stage in the development of thyroid cancer, which was ahead of the existing clinical diagnostic methods such as cytopathology and histopathology. At present, no signs of recurrence or metastasis were observed during follow-up (6 months) in two patients whose tissues were confirmed to be benign after surgery. The early prediction of ARHI imprinted gene status change is thyroid cancer, but this still needs to be confirmed by evaluation of large samples.

Compared with the traditional detection method FNAC, the consistency test Kappa value of ARHI imprinted gene detection was 0.707, with a significant difference; the AUC values of the two methods were 0.850, indicating that the imprinted gene detection had a good agreement with FNAC in the diagnosis of thyroid benign and malignant tumors, and they had similar diagnostic value. However, ARHI imprinted gene detection had a higher sensitivity (100%). In terms of detection rate, in 35 cases of puncture, the detection rate of FNAC was 85.7%, while that of ARHI imprinted gene detection was 91.4%. In addition, the malignancy detection rate of ARHI imprinted gene was 100% (all cases confirmed to be malignant by postoperative pathology were determined positive by imprinted gene), while the malignancy detection rate of FNAC was 82%. There were no significant differences in the specimens between the two methods because the samples were taken from the same lesion by multi-needle puncture. In the process of specimen preparation, imprinted gene detection was performed by directly injecting the specimen into cell lysate, which was far less skillful than FNAC smear preparation. In the process of reading the specimen, the total expression amount, LOI, and CNV of imprinted genes in a single cell were visually observed by imprinted gene diagnosis *in situ*, which was objective and not affected by the doctor's proficiency (Wei and Wang, 2016).

It is worth noting that the results of FNAC in patients with FTC confirmed by postoperative pathology in this study were benign; the reason was that there were some overlaps to a certain extent in the morphological manifestations of benign and malignant thyroid lesions originated from follicular cells, cytopathology could not reflect the overall picture of the tumor and the interrelation between the tumor and surrounding tissues, and it was almost impossible to differentiate microinvasive follicular carcinoma from benign follicular adenoma, eosinophilic adenoma, and oncocytic carcinoma in cytology (Gürkan *et al.*, 2013; Fang *et al.*, 2015). In the endocrine tumor WHO classification published in 2017, “follicular tumor with undetermined malignant potential,” “highly differentiated tumor with undetermined malignant potential,” and “follicular tumor with noninvasive papillary carcinoma nuclear characteristics” were newly diagnosed as thyroid tumors, which were three borderline lesions with uncertain benign and malignant (Liu *et al.*, 2018); these three types of lesions could hardly be diagnosed by cytopathological examination alone, causing great trouble for the follow-up clinical intervention. Contrary to the results of FNAC, the results of imprinted gene detection in FTC patients were malignant, which was related to the different principles of the two detection methods, suggesting that ARHI imprinted gene detection has good diagnostic value for such borderline lesions that are difficult to be defined as benign and malignant.

This study was a single-center study, the sample size was small, and the malignant proportion of thyroid nodules in the selected population was large, and a few patients' pathological types were not confirmed by surgery; these factors may cause some bias to the results. Although imprinted gene detection has advantages in the diagnosis of follicular tumors, whose biological behavior are difficult to determine, it still needs to be evaluated by large samples. In 2009, BSRTC was established by the American Institute of International Oncology to classify the thyroid FNAC results in a more standardized way (Sullivan *et al.*, 2014). In this study, cell diagnosis was still based on the classification criteria of 2002, and there was a certain bias for the results, especially for malignant potential, whose malignancy rate was only 60%, significantly lower than the recommended range of SM in BSRTC (Krauss *et al.*, 2016; Krooks *et al.*, 2018; Lanfranchi *et al.*, 2018). Therefore, the application value of the above two methods in the differential diagnosis of benign and malignant thyroid nodules still needs to be verified in subsequent clinical practice.

In conclusion, there are no significant differences between FNAC and imprinted gene detection in the differential diagnosis of benign and malignant thyroid, and imprinted gene detection has higher sensitivity and accuracy. *In situ* detection of imprinted genes as a new diagnostic technology may provide accurate diagnosis and favorable therapeutic opportunities for early-stage cancer patients.
